# Layering Optimization of the SrFe_0.9_Ti_0.1_O_3−δ_–Ce_0.8_Sm_0.2_O_1.9_ Composite Cathode

**DOI:** 10.3390/molecules27082549

**Published:** 2022-04-14

**Authors:** Azreen Junaida Abd Aziz, Nurul Akidah Baharuddin, Mahendra Rao Somalu, Andanastuti Muchtar

**Affiliations:** 1 Fuel Cell Institute, Universiti Kebangsaan Malaysia, Bangi 43600, Selangor, Malaysia; p102346@siswa.ukm.edu.my (A.J.A.A.); mahen@ukm.edu.my (M.R.S.); muchtar@ukm.edu.my (A.M.); 2 Department of Mechanical & Manufacturing Engineering, Faculty of Engineering and Built Environment, Universiti Kebangsaan Malaysia, Bangi 43600, Selangor, Malaysia

**Keywords:** area-specific resistance, electrochemical impedance, layered structures, microstructures, solid oxide fuel cell

## Abstract

Cathode thickness plays a major role in establishing an active area for an oxygen reduction reaction in energy converter devices, such as solid oxide fuel cells. In this work, we prepared SrFe_0.9_Ti_0.1_O_3−δ_–Ce_0.8_Sm_0.2_O_1.9_ composite cathodes with different layers (1×, 3×, 5×, 7×, and 9× layer). The microstructural and electrochemical performance of each cell was then explored through scanning electron microscopy and electrochemical impedance spectroscopy (EIS). EIS analysis showed that the area-specific resistance (ASR) decreased from 0.65 Ωcm^2^ to 0.12 Ωcm^2^ with the increase in the number of layers from a 1× to a 7×. However, the ASR started to slightly increase at the 9× layer to 2.95 Ωcm^2^ due to a higher loss of electrode polarization resulting from insufficient gas diffusion and transport. Therefore, increasing the number of cathode layers could increase the performance of the cathode by enlarging the active area for the reaction up to the threshold point.

## 1. Introduction

Layering mechanism optimization is known to play an important role in composite-related fields [1,2]. The layered structure is also prominently used in energy converter devices (e.g., solid oxide fuel cell (SOFC)). SOFCs show potential for future application in supplying electricity via chemical reaction without any combustion. Therefore, it is a green technology and highly efficient in providing electricity. A large number of SOFCs have been commercialized in the form of combined heat and power plants, but they remain in the design stage because of high operating temperatures, which are generally approximately 800 °C to 1000 °C. The critical challenges of SOFC development are high cost and low performance because they are used at high temperatures [3]. Reducing the operating temperature of SOFCs can provide remarkable advantages and help commercialize this technology faster. Intermediate-temperature SOFC (IT-SOFC) and low-temperature SOFC (LT-SOFC) offer a reduction in material costs. Accordingly, the costs of SOFCs can be minimized. However, reducing the operating temperature also causes several issues; for instance, the activation concentration increases and contributes to ohmic polarization, which affects the SOFC performance. Components that can excel at lower temperature ranges should be selected and constructed to reduce these problems. These problems are resolved by using certain methods, such as reducing electrolyte thickness and creating a new material with an increased oxygen ion conductivity [4].

Studies have focused on the effects of increasing electrode thickness to overcome this problem [5,6]. Fang et al. simulated the influence of layer thickness on the structural integrity of SOFCs; they found that the proportion of compressive stress–strength at the cathode decreases with the increase in cathode thickness [7]. Abdul Samat et al. showed that the difference in cathode thickness affects the electrochemical performance of symmetrical cells because of the different sizes of the active area in the cathode when the cathode thickness increases or decreases [8]. Abdul Samat et al. concluded that increasing the cathode film thickness to a certain level enlarges the reaction area and improves the electrochemical reaction activity of cathodes. Another method to lower the SOFC working temperature is by developing new materials. Baharuddin et al. discarded cobalt from an SOFC material to prevent delamination between a cathode and an electrolyte through thermal mismatch reduction [9]. They used a strontium-based material (SrFeTiO_3−δ_) to discard cobalt in the cathode of IT-SOFC [10]. Cobalt can also create a large thermal expansion coefficient (TEC) that can lead to the delamination of the components in SOFCs [11]. Some new materials with a high electron and ion conduction have also been introduced to lower the temperature throughout their 15 years of effort in studying new materials for IT-SOFC and LT-SOFC [12]. Electrolyte materials have also been added to a cathode material to form a composite cathode material [13] to help increase the thermal expansion coefficient between electrolytes and electrodes.

Reduced losses of ohmic polarization can be accomplished by creating new effective materials with strong ionic conductivity. Examples of ionic-conductivity materials are gadolinium-doped ceria (GDC), samarium-doped ceria (SDC), and scandia-doped zirconia (SDZ) electrolytes. In addition to ohmic polarization loss reduction, polarization losses in the cathode materials, especially those involving the activation and concentration, should be minimized to produce SOFCs with optimum performance at relatively low operating temperatures. A significant loss of the voltage occurs while reducing a temperature SOFC activity because of the losses of the activation polarization at the cathode, directly affecting the overall output of SOFCs [14]. Reduced operating temperatures increase the level of energy activation of the oxygen reduction reaction (ORR) and oxide ion transfer in cathodes; accordingly, this mechanism is considered the primary rate-determining stage of SOFC processing at reduced temperatures [15]. Therefore, cathode material development should be intensively studied to decrease the working temperature of SOFCs. The primary objective of an SOFC cathode is to provide functional areas for oxygen molecule reaction, such as reduction to become oxygen ions. The oxygen ions will eventually transfer from the cathode side to the electrolyte side [16]. The chemical structure, durability, and electrochemical performance will be examined in selecting the materials for SOFC cathodes. The oxide phase with an ABO_3_ perovskite-structured material is preferable as an effective material for cathode IT-SOFC due to its favorable electrochemical behavior in a reduction scenario [17]. In particular, SrFeTiO_3−δ_ has been widely explored due to its mixed ionic–electronic conductivity (MIEC) activity and strong ionic and electronic conductivity [18].

In this work, SrFe_0.9_Ti_0.1_O_3−δ_ (SFT) as a new cathode material was mixed with SDC as an electrolyte material to become a composite cathode. SDC, a commonly used electrolyte with a high-performance record [19], was mixed with the main cathode material to reduce the TEC between the cathode and the electrolyte. This procedure avoided delamination and extended the life of SOFCs. Then, the cathode composite SFT–SDC was manually printed in a multilayered structure to form a multilayered SFT–SDC composite cathode. The performance of this multilayered SFT–SDC was evaluated in terms of electrochemical performance versus number of layers. The layer printed on SDC varied from one layer to nine layers to maximize the thickness of the thin-film cathode printed on the substrate (electrolyte).

## 2. Materials and methods

### 2.1. Sample Preparation

Ce_0.8_Sm_0.2_O_1.9_ (SDC) commercial powder (Sigma-Aldrich, St. Louis, MO, USA) was used to fabricate an electrolyte pellet. A button pellet (25 mm diameter) of SDC was pressed with a hydraulic press machine (Carver Inc., Wabash, Indiana, USA) with a pressure of 5.2 tons for a holding time of 1 min. The press SDC pellet was calcined at 1400 °C for 6 h. This button pellet SDC was used as an electrolyte. A powder of SFT was produced via glycine nitrate combustion. Sr(NO_3_)_2_ and Fe(NO_3_)_3_·9H_2_O were stirred for 45 h with the presence of de-ionized water and TiO(NO_3_)_2_. All powders were purchased from Sigma-Aldrich. Stoichiometric ratio for the SFT reaction is Sr(NO_3_)_2_ + 0.9Fe(NO_3_)_3_·9H_2_O + 0.1TiO(NO_3_)_2_ + *y*NH_2_CH_2_COOH to SrFe_0.9_Ti_0.1_O_3−δ_ + *A*N_2_ + *B*CO_2_ + *C*H_2_O. The precursor powder appeared after the combustion of dark ash. The dark ash was heated (calcined) at 1300 °C to achieve the desired SFT powders. A powder of SFT and SDC was mixed at a 9:1 ratio, forming 9SrFe_0.9_Ti_0.1_O_3−δ_–1Ce_0.8_Sm_0.2_O_1.9_ (9SFT-1SDC). Afterward, it was mixed with acetone as a binder and placed in a ball mill with a high-energy operation at 250 rpm for 2 h. The slurry of the 9SFT-1SDC cathode was made by using a roll mill machine with a triple roller (EGM-65, ELE, Shanghai, China). At this stage, terpinol was used as a solvent, ethyl cellulose was utilized as a binding agent, and hypermer KD15 (Croda, Snaith, UK) was set as a dispersant to make a slurry. A manual print screen technique was applied to print a layer of 9SFT-1SDC cathode ink on the SDC pallet surface. One layer (1×), three layers (3×), five layers (5×), and nine layers (9×) of the cathode ink were printed on the SDC at both sides to form a symmetrical 9SFT-1SDC/SDC/9SFT-1SDC cell and evaluate the cathode thickness and layer effect. The cathode was consistently printed at a size of 1 cm^2^ on both sides of the electrolyte. Subsequently, the cell was dried before the next layer was printed. After the desired layer was formed, the symmetrical cell was heated (sintered) at 1250 °C for 2 h.

### 2.2. Sample Characterization

The cross-sectional image of the different layer cathode print was obtained with a scanning electron microscope (SEM, Zeiss, Oberkochen, Germany) to evaluate the morphological characteristics and thickness of the 9SFT-1SDC/SDC/9SFT-1SDC symmetrical cell. Image recognition tools (ImageJ) were utilized to investigate the surface morphology, such as the particle size of the cathode thin film. The thickness of the cathode film was measured with an SEM when the image was being captured. Electrochemical impedance was measured with the potentiostat at a working temperature of 800 °C with an airflow of 200 mL/min and a current of 0.001 A. The analysis of the electrochemical impedance was fitted by using NOVA 1.0. Real impedance (Z′) versus imaginary impedance (Z″) was plotted with the OriginLab 2019b version. Area-specific resistance was calculated using Equation (1):

ASR = (*R_p_* × A)/2, (1)

where

(2) $$R_{p}=\left(R_{1}+R_{2}\right),\;$$

where *R_p_* is the interfacial cathode and electrolyte polarization resistance. $R_{1}$ is the initial high-frequency arc produced by the charge transfer process associated with the integration of an O^2−^ ion through the SFT-SDC composite and at the SFT-SDC composite cathode/SDC electrolyte interface. $R_{2}$ is the second low-frequency arc associated with the dissociation/absorption of oxygen molecules and the diffusion process at the SFT-SDC cathode surface. A is the cathode’s area of activity. In this case, the composite 9SFT-1SDC active area is consistently printed at 1 cm^2^ for all symmetrical cells. Therefore, the value is constant at 1 cm^2^.

## 3. Result and Discussion

### 3.1. Microstructure of the Fabricated Pellet

Figure 1 displays the X-ray diffraction (XRD) patterns of the 9SFT-1SDC composite powders. The composite cathodes are assignable to two perovskite phases of SrFe_0.9_Ti_0.1_O_3−δ_ and SDC. No remarkable secondary phase from the resultant 9SFT-1SDC powder is detected within the XRD sensitivity. The introduction of SDC into SFT does not influence its structure as the composite cathode powders are able to maintain their own structure after mixing.

The cross-sectional micrograph of 9SFT-1SDC was obtained via SEM. Figure 2 shows the micrograph of 9SFT-1SDC with (a) one layer (1×), (b) three layers (3×), (c) five layers (5×), (d) seven layers (7×), and (e) nine layers (9×). The SDC electrolyte fabricated at 1400 °C is highly dense from the micrograph pictures of all five structures. Hussain et al. demonstrated that a good SDC electrolyte should be dense enough to stop the movement of gas passing through the electrolyte layer. The development of the SDC electrolyte demonstrated high ionic conductivity at low temperatures of 400 °C–600 °C, a capacity to produce oxygen ions at comparable temperatures, and chemical stability, which are desirable properties for LT-SOFCs [20]. Accordingly, we chose SDC as an electrolyte for this study because it has been proven to be a good electrolyte with an ABO_3_ cathode.

The layer was observed in the micrograph images with a transparent barrier between the cathode and the electrolyte layers. However, the cathode layer separately printed and dried using an oven could not be detected. It appeared as a single-layer cathode with variations in thickness only. Overall, the 9SFT-1SDC cathode showed a clear change in thickness by increasing the number of layers.

All five symmetrical cells exhibited a good adhesion to the electrolytes. The thicknesses of one-, three-, five-, seven-, and nine-layer cathodes were measured at 6.86 (1×), 13.40 (3×), 19.54 (5×), 25.60 (7×), and 30.95 µm (9×), respectively, through SEM measurement. The error bar was added to the figure as the thickness measurement was conducted eight times for each sample to show the distribution of the thickness values. The thickness slope gradually increased at a 3.02 μm ± 0.04 μm increment with the increase in the number of printed layers as shown in Figure 3. From the figure, one can see that the extrapolation leads to a positive *y*-intercept at 4.12 μm ± 0.24 μm. This contradiction is probably because of a slight difference in the applied pressure during the manual printing process. In this work, the applied pressure is assumed to be constant during the deposition of each layer onto the electrolyte substrate.

The surface porosity of the 9SFT-1SDC cathode microstructure was captured using public domain software ImageJ, software version 1.53a, National Institutes of Health, USA, for the estimation of porosity (Figure 4). The best porosity of the cathode SOFC should vary at approximately 20% to 40% [21]. Oxygen diffusion efficiently works with this range of porosity. It provides enough room for oxygen to diffuse to the electrolyte. Baharuddin et al. [6] showed the increment in porosity by increasing the number of layers. However, in this study, porosity increased only from one layer to five layers and then decreased as the number of layers increased from seven to nine layers.

This phenomenon is likely attributed to the strength applied while manually printing the cathode layers on the electrolyte. The hand-press applied to the squeegee while printing the cathode layer stressed the material, causing it to form a pile that became denser with the increase in the thickness of the film’s cathode. When the cathode film thickness was increased during printing, the latest layer was close to the print screen, thereby reducing the gap while printing the next layer. Accordingly, this phenomenon increased the load applied to the next layer. The illustration of this phenomenon is shown in Figure 5 for a better understanding. The changes in the gap between the cathode film and the mesh can be observed in illustrations (b) to (d). The reduced printing gap made the film denser, whereas the hand load applied was also another uncontrollable parameter in manual film printing. Somalu et al. explained that the squeegee-applied load, squeegee rate of speed, design of the squeegee, type of screen mesh, and distance for the snap-off (distance gap between the screen mesh and substrate) of the screen printer are important criteria for the output of good-quality films. Additionally, their analysis indicated that the thickness of the studied YSZ film decreased when the squeegee load increased [22].

Another factor is the thicker layer embedded on the layer, which compresses the bulk cathode ink and causes the microstructure to become denser. Accordingly, the seven and nine layers of the cathode were found to have reduced porosity. Such a phenomenon occurred when a manual print screen was employed in printing the film layer because the human factor affected the thickness consistency of the film. This finding likely occurred because the squeegee pressure could not be set at a certain number when the manual print screen technique was used. Somalu et al. [23] showed a consistent layer of cathode film printing when a consistent squeegee pressure was applied by employing a print screen machine.

### 3.2. Electrochemical Reaction of the Fabricated Pellet

The effects of film thicknesses, especially on the polarization resistance of the composite cathode 9SFT-1SDC, were studied. The 9SFT-1SDC was fabricated as a symmetrical cell of various thicknesses, and its electrical output was evaluated at 800 °C. An equivalent circuit model of *R_s_*(*R_1_*CPE_1_)(*R_2_*CPE_2_) was used to satisfy the whole EIS spectrum at 800 °C. *R_s_* is the ohmic resistance of the electrolyte SDC. *R_1_* would be the first curve at a high frequency caused by the process of charge transfer related to the integration of O^2−^ via the 9SFT-1SDC composite cathode and at the 9SFT-1SDC composite cathode and the interface of the SDC electrolyte. *R_2_* is the curve at a low frequency caused by the dissociation/adsorption of O^2−^. CPE_1_ and CPE_2_ refer to the constant-phase components.

The EIS spectrum was plotted (Figure 6) to evaluate the efficiency of the prepared symmetrical cells. The equivalent circuit was also added in the lower right corner in Figure 6. *R*_1_ was fully reliant on the 9SFT-1SDC thickness, indicating that the 9SFT-1SDC composite thickness significantly affected the transfer of charge mechanism related to the high-frequency curve. Even then, *R*_2_ decreased in response to changes in the thickness of the 9SFT-1SDC cathode. The 9SFT-1SDC composite cathodes could serve as an active site for the ORR from the interface to the TPB, and several routes for O^2−^ migration to the electrode and electrolyte interface. The overall ASR of the different thicknesses of the 9SFT-1SDC composite cathode slightly varied due to the cumulative effects of *R*_1_ and *R*_2_. The cathode ORR was composed of multiple stages at varying time constants: (1) oxygen adsorption and desorption on the cathode surface, (2) dissociation of the oxygen being adsorbed, (3) ionization of the adsorbed oxygen, (4) surface diffusion of the adsorbed oxygen, (5) ionic conduction of the adsorbed oxide ion in the bulk cathode, and (6) charge transfer of the adsorbed oxide ion at the electrode/electrolyte interface [24].

The electrochemical reaction occurs at the cathode’s triple-phase boundary (TPB), which is formed by the cathode, electrolyte, and gas phase [25]. At the electrode and electrolyte connection boundaries, the electrochemical reaction that occurred at the cathode area is aligned with the reaction associated with the adsorbed oxygen molecules and reaction of electrons to form O^2−^ [26]. The Kröger–Vink notation can be used to express this reaction:

(3) $$\frac{1}{2}\;O_{2}+2e^{-}+V\ddot{o}\to O_{o}^{x},$$

where $V\ddot{o\;}$ is the vacancy of the oxygen species in the cathode, $e^{-}$ is the cathode electron, and $O_{o}^{x}$ is the oxide ion. ORR occurs in the MIEC composite cathode at the three- and two-phase boundaries between the MIEC and the gas phase [27]. Accordingly, 9SFT-1SDC, as an MIEC, also forms a high three-phase boundary with a two-phase boundary and obtains a high ORR activity. After the insertion of the SDC electrolytes into the SFT cathode, the reaction described in Equation (4) may be carried out using $V\ddot{o\;}$ from *SDC*, where $O_{o}^{x}$ of *SDC* is the lattice oxygen in *SDC* [3]:

(4) $$O_{o}^{x}\left(SDC\right)+V\ddot{o}\left(SFT\right)\to \;O_{o}^{x}\left(SFT\right)+V\ddot{o}\left(SDC\right).\;$$

The reaction expressed in Equation (4) occurs at the boundaries of the surface 9SFT-1SDC composite cathode where the gas phase reaches. At triple-phase boundaries, the oxygen integration reaction is measured by the number of oxygen molecules adsorbed to the 9SFT-1SDC surface in Equation (4) and the oxygen vacancy amount as captured by the chemical reaction described in Equation (5):

(5) $$O_{ad}^{2^{-}}\left(2PB\right)+V\ddot{o}\left(SDC\right)\to \;O_{o}^{x}\left(SDC\right).\;$$

The amount of $V\ddot{o}\left(SDC\right)$ is critical in determining the successful ORR in the 9SFT-1SDC composite cathode, especially the reaction involving the kinetic surface exchange and rate of bulk oxygen transport. This parameter is translated into a number via the ASR test. The number of electrochemically active sites grew as the 9SFT-1SDC thickness increased up to seven layers of film printing.

Abdullah et al. also showed a decrease in the ASR in their experiment by using the LSC cathode at a thin cathode layer because of the insufficient active area. They increased the cathode layer up to 8× and obtained optimum ASR values. When the layer increased to 8×, the ASR was higher than that starting at the 2× layer [8]. The same result was derived in this study, where the ASR values decreased with the increase in the thickness by adding the number of layers. When the number of the cathode layers increased, *Rp* decreased to seven layers. The 7× layer provides optimum values of a good ASR at 0.12 Ωcm^2^. However, the values greatly increased when the 9× cathode prints to 2.95 Ωcm^2^. This is believed due to the lowest porosity (13.98%) shown by the 9× cathode layer. The porosity of the cathode determines how well molecular oxygen can permeate it and reach the active sites, as well as how well oxide ions can diffuse from the point of incorporation into the MIEC lattice to the cathode/electrolyte interface. The thickness of the film also increases the reaction area for the oxide to diffuse to the cathode/electrolyte interface. The total TPB length available for the reaction within the cathode is low in thin electrodes, so oxygen reduction is limited by a lack of reacting sites, resulting in a high area of specific resistance. While thick cathodes are less conductive, even though they have a longer TPB length (though the TPB per unit volume is lower locally), cathode performance is limited by charge transport. The result is illustrated in Table 1.

Increasing or decreasing the thickness of the electrode has a dynamic effect on the kinetics of this operation. The surface area increases by augmenting the thickness of the electrode. Accordingly, the number of possible areas for the absorption and dissociation of oxygen molecules increases. This result promotes the kinetic mechanism of molecular oxygen absorption and dissociation on the surface accompanied by the diffusion of dissociated oxygen species on the surface [28]. Simultaneously increasing the electrode thickness has a detrimental effect. The oxygen species that are not related to either charged or uncharged oxygen atoms must migrate to the catalytically active region through surface diffusion, through which they are ionized and integrated into the lattice [29]. The diffusion or distribution length of these oxygen species is increased by increasing the thickness of the electrode.

## 4. Conclusions

A composite cathode composed of 9SFT and 1SDC was successfully fabricated in this work through glycine nitrate combustion and assisted through high-energy ball milling for a composite well mixture. The 9SFT-1SDC composite cathode with seven layers of printing with a film thickness of 25.60 µm had a low ASR at 0.12 Ωcm^2^, indicating the good performance of the cathode. This value broadened the activity areas with an electrochemical reaction compared with the rest of ASR with different layers (1×, 3×, 5×, 7× and 9×). Accordingly, seven layers of thickness at approximately 25 µm could be considered the optimum active area for 9SFT-1SDC materials. Therefore, the thickness of the cathode may be adjusted to optimize its electrochemical properties and the efficiency of the symmetric cathode cells.

## Figures and Tables

**Figure 1:** X-ray diffraction patterns of the fabricated 9SFT-1SDC composite cathode, SFT and SDC.

**Figure 2:** SEM images of the cross-section of (**a**) 1× printing, (**b**) 3× printing, (**c**) 5× printing, (**d**) 7× printing, and (**e**) 9× printing. EDX image is for powder 9SFT-1SDC.

**Figure 3:** Thickness of 9SFT-1SDC composite cathode deposited on SDC electrolyte.

**Figure 4:** Porosity for (**a**) 1× printing, (**b**) 3× printing, (**c**) 5× printing, (**d**) 7× printing, and (**e**) 9× printing calculated using ImageJ software.

**Figure 5:** Illustration of the print screen with manually applied load. (**a**) Overall setup for the cathode film printing, (**b**) 1× printing, (**c**) 3× printing, and (**d**) 5× printing.

**Figure 6:** Nyquist plot (impedance spectrum) of the symmetric 9SFT-1SDC cells with 1×, 3×, 5×, 7×, and 9× layer printing and the equivalent circuit.

**Table 1:** Number of layers with film thickness, ASR, and porosity.

Symmetrical Cell	Number of Layers	Film Thickness (µm)	Porosity (%)	ASR (Ωcm^2^)
9SFT-1SDC (1×)	1	6.42	21.52	1.25
9SFT-1SDC (3×)	3	13.40	23.00	0.65
9SFT-1SDC (5×)	5	19.54	25.59	0.22
9SFT-1SDC (7×)	7	25.60	22.87	0.12
9SFT-1SDC (9×)	9	30.95	13.98	2.95

## Data Availability

Not applicable.

## Sample Availability

Samples of the compounds SFT and SDC are available from the authors.
